The article "Transnasal High-Flow Oxygen Therapy versus Noninvasive Positive Pressure Ventilation in the Treatment of COPD with Type II Respiratory Failure: A Meta-Analysis" was retracted in 2023. Reasons: signs of a paper mill; suspected computer-generated content; unreliable results or conclusions; concerns about the data.

# Transnasal High-Flow Oxygen Therapy versus Noninvasive Positive Pressure Ventilation in the Treatment of COPD with Type II Respiratory Failure: A Meta-Analysis

**DOI:** 10.1155/2022/3835545

**Published:** 2022-07-26

**Authors:** Wei Liu, Mingli Zhu, Liuqin Xia, Xiangying Yang, Pei Huang, Yanming Sun, Ye Shen, Jianping Ma

**Affiliations:** ^1^Zhejiang Chinese Medical University, Hangzhou, Zhejiang, China; ^2^Department of Critical Care Medicine, Affiliated Hangzhou First People's Hospital, Zhejiang University School of Medicine, Hangzhou, Zhejiang, China

## Abstract

**Objective:**

To compare the safety and efficacy of transnasal high-flow oxygen therapy (HFNT) and noninvasive positive pressure ventilation (NIV) in the treatment of chronic obstructive pulmonary disease (COPD) with type II respiratory failure.

**Methods:**

PubMed, the Cochrane Library, Embase, CBM, CNKI, and other databases were searched for randomized controlled trials (RCTS) on the efficacy of HFNT and NIV in the treatment of COPD. Meta-analysis was conducted using RevMan 5.3 software after two researchers screened literatures, extracted data, and evaluated the methodological quality of the included studies according to inclusion and exclusion criteria.

**Results:**

A total of 948 patients were included in 12 RCTS. Comprehensive analysis results showed that the HFNC group had higher levels of 12 h-PAO_2_, 48 h-PACO_2_ and, 48 h-pH than the NIV group, and the differences were statistically significant (*P* < 0.05). There were no significant differences in 24 h-PAO_2_ and 72 h-PAO_2_, 12 h-PACO_2_, 24 h-PACO_2_ and 72 h-PACO_2_, 24 h-pH, 48 h-pH, and 72 h-pH between the two groups after treatment (*P* > 0.05).

**Conclusions:**

Compared with NIV, HFNC does not increase the treatment failure rate in COPD patients with type II respiratory failure, and HFNC has better comfort and tolerance, which is a new potential respiratory support treatment for COPD patients with type II respiratory failure.

## 1. Introduction

Chronic obstructive pulmonary disease (COPD) is a common, preventable, and treatable disease characterized by persistent respiratory symptoms and restricted airflow due to abnormalities in the airways and/or alveoli [1]. The prevalence of COPD is rapidly increasing and is going to become the third leading fatal disease in the world by 2030 [2]. COPD is characterized by progressive, irreversible airflow restriction and is resource-efficient and costly due to outpatient visits, chronic treatment, and frequent hospitalizations for the disease. Chronic hypercapnia respiratory acidosis is a common feature of acute exacerbation of COPD, which is called acute hypercapnia respiratory failure (AHRF) [3]. At this time, severe ventilation dysfunction occurs in the patient, and the probability of disability and death is very high if the patient does not receive timely and effective treatment [4]. Clinically, emergency endotracheal intubation assisted by an invasive ventilator can significantly improve the respiratory status of patients, but there are still some cases after extubation, such as incomplete control of pulmonary infection, weak muscle strength, poor expectoration ability, and mild respiratory failure, which require postextubation treatment. Traditional oxygen therapy has poor effect on the treatment of humidification after extubation, which is easy to cause dry sputum and difficult to cough up, which is not conducive to improving respiratory failure [5].

Nearly half of COPD patients with AHRF did not survive in the first year after target hospitalization, 80% required readmission, and nearly two-thirds had another life-threatening event [6]. In the case of AHRF, the unique optimization failure of standard drug therapy may be as high as 74%. In addition to drug therapy, the 2019 guidelines showed that the success rate of noninvasive ventilation (NIV) in treating COPD was 80%~85% [7]. NIV refers to a ventilation application without any conduit into the airway, that is, without an endotracheal tube or tracheostomy tube. NIV improves vital signs and gas exchange, increases alveolar ventilation, and reduces dyspnea, intubation needs, length of ICU stay, and mortality. NIV, however, may not be well tolerated, and about 25% of subjects have NIV contraindications [8]. The high-flow nasal cannula (HFNC) is used to enhance ventilation while providing higher oxygen concentration. HFNC uses a fully regulated, heated, and humidified air/oxygen mixture to give oxygen to patients through large-caliber nasal cannula at a flow rate of 20-60 L/min [9]. HFNC reduces anatomic dead space in the nasopharyngeal airway, improves mucociliary clearance in the great bronchus and small trachea, and increases end-expiratory pressure. HFNC forms a significant blood-dependent CO_2_ flushing effect in nasopharyngeal space, which can reduce ventilation of anatomic dead space and thus reduce CO_2_ retention [10]. Additional evidence in lung rehabilitation suggests that HFNC as part of rehabilitation training may improve exercise endurance in patients with COPD as opposed to conventional oxygen therapy, but further studies are needed to evaluate the efficacy of the therapy. Oxygen intake during exercise training allows COPD patients to tolerate higher activity levels and reduce fatigue symptoms, ultimately improving their quality of life.

Both HFNC and NIV can improve the respiratory pattern of hypercapnia patients during COPD exercise training to varying degrees by measuring diaphragm pressure, respiratory pattern, and gas exchange, which may play a role in the long-term treatment of patients. For patients with hypoxemic COPD, exercise training can effectively improve exercise capacity and there may be differences in oxygen therapy. At present, regarding the efficacy of HFNC and NIV, we still need to investigate whether all patients can benefit from NIV or HFNC treatment, and this study explored this question.

## 2. Materials and Methods

### 2.1. Data Retrieval

Two researchers screened articles by reading abstracted data published in the database until October 2021 to compare randomized controlled trials (RCTs) of the HFNC group and NIV group in the treatment of COPD with hypercapnia. Specific retrieval methods: PubMed, Cochrane Library, Embase, CBM, CNKI, and other databases were searched. Search using MeSH terms and test words: high flow or high-flow or noninvasive or non-invasive and COPD or chronic obstructive pulmonary disease. The type of literature was limited to RCTs and included only adult patients over 18 years of age. References to all relevant studies and recent review articles were scanned to identify additional citations. After the exclusion of obviously irrelevant publications, further full-text screening of potentially eligible articles is carried out according to our predefined inclusion criteria, and disagreements are resolved by consensus.

### 2.2. Inclusion Criteria

Twelve RCTs were included in this study. Subjects were COPD patients with acute respiratory failure complicated by hypercapnia according to the guidelines for chronic obstructive pulmonary disease [11], and the blood gas analysis results after admission were arterial partial blood oxygen pressure (PaO_2_ < 60 mmHg) and arterial partial pressure of carbon dioxide (PaCO_2_ < 50 mmHg). All the articles were related to the NIV group and HFNC group. The observation indexes included blood gas indexes such as PaO_2_, PaCO_2_, hydrogen ion concentration index (pH), and the incidence of complications.

### 2.3. Exclusion Criteria

The exclusion criteria were as follows: under the age of 18; severe respiratory failure requiring immediate endotracheal intubation: respiratory rate >40 times/min; severe hypoxia (oxygenation index under high concentration of oxygen inhalation < 150 mmHg, severe respiratory acidosis pH < 7.25, disturbance of consciousness, etc.); NIV contraindications exist, including oral and facial trauma, excessive sputum and poor sputum discharge ability, and hemodynamic instability, etc.; poor short-term prognosis; increased risk of death within 7 days; ongoing palliative care; failure of other organs; tracheotomy; poor treatment compliance; no comparison between the two groups; incomplete information; and not meeting inclusion criteria.

### 2.4. Quality Evaluation of the Included Literature

The quality of the included literature was evaluated independently by two researchers according to the Cochrane Review Manual. The evaluation contents include the following: (1) random allocation method, (2) hidden allocation scheme, (3) blind method, (4) completeness of outcome indicators, (5) selective reporting, and (6) other sources of bias. The literature was graded according to the evaluation results. Grade A is when a patient fully meets the above criteria, with low risk of bias; partially meeting the above criteria belongs to grade B, with moderate risk of bias; and completely not meeting the standard is grade C, indicating a high risk bias. For literatures with inconsistent opinions, a third party shall intervene and negotiate to determine the quality of literatures.

### 2.5. Data Extraction and Statistical Processing

Basic information includes first author, year of publication, treatment of COPD, and number of cases. The observation indexes included blood gas analysis and complication indexes, such as PaO_2_, PaCO_2_, and pH. Statistical data were extracted using the RevMan 5.3 software package. Relative risk and 95% CIs were used for dichotomy data, standard mean difference and 95% CIs were used for continuous data, and funnel plots were used to assess publication bias at test level *α* = 0.05.

## 3. Results

### 3.1. Retrieval Results and Risk of Bias

According to the predefined retrieval strategy, a total of 12 RCTs [12–23] were screened out, and 948 RCTs were reviewed from the bias risk review. A total of 473 patients were treated with a noninvasive ventilator, and 475 patients were treated with high-flow humidified oxygen therapy (Fisher Pike, New Zealand) (Figure 1).

### 3.2. Comparison of 12 h-PaO_2_ after Treatment between the HFNC Group and NIV Group

Four studies [13, 14, 17, 20] reported 12 h-PAO_2_, with no heterogeneity between studies (*P* = 0.82, *I*^2^ = 0%). The fixed effects model was used for analysis, and the difference between the two groups was statistically significant (SMD = 0.47, 95% CI (0.26, 0.68), *P* < 0.0001), and the HFNC group had an advantage in the treatment of 12 h-PAO_2_ in acute respiratory failure (Figure 2).

### 3.3. Comparison of 12 h-PACO_2_ after Treatment between the HFNC Group and NIV Group

Four studies [13, 14, 17, 20] reported 12 h-PACO_2_, with interstudy heterogeneity (*P* < 0.00001, *I*^2^ = 90%), which was analyzed using a random effects model. The results showed that there was no significant difference between the two groups (SMD = 0.15, 95% CI (-0.52, 0.83), *P* = 0.66) (Figure 3).

### 3.4. Comparison of 24 h-PAO_2_ after Treatment between the HFNC Group and NIV Group

Eight studies [12–14, 16, 18, 19, 21, 23] compared 24 h-PaO_2_ in the HFNC group and NIV group. There was no significant difference in heterogeneity among studies (*P* = 0.14, *I*^2^ = 37%), and the fixed effects model was used for analysis. The results showed that there was no significant difference between the HFNC group and NIV group (SMD = 0.08, 95% CI (-0.08, 0.25), *P* = 0.31) (Figure 4).

### 3.5. Comparison of 24 h-PACO_2_ after Treatment between the HFNC Group and NIV Group

Nine studies [12–14, 16, 18, 19, 21, 23] compared 24 h-PACO_2_ in the HFNC group and NIV group. There was no significant difference in heterogeneity among studies (*P* = 0.62, *I*^2^ = 0%), and the fixed effects model was used for analysis. The results showed that there was no significant difference between the HFNC group and NIV group (SMD = −0.05, 95% CI (-0.21, 0.11, *P* = 0.53) (Figure 5).

### 3.6. Comparison of 24 h-pH after Treatment between the HFNC Group and NIV Group

Seven studies [13, 14, 16, 18, 19, 21, 23] reported 24 h-pH with interstudy heterogeneity (*P* = 0.001, *I*^2^ = 6%) and were analyzed using a random effects model. The results showed that there was no significant difference between the HFNC group and NIV group (SMD = 0.13, 95% CI (-0.25, 0.1), *P* = 0.86) (Figure 6).

### 3.7. Comparison of 48 h-PAO_2_ after Treatment between the HFNC Group and NIV Group

Five studies [16–18, 21, 23] compared 48 h-PAO_2_ in the HFNC group and NIV group. There were statistically significant differences in heterogeneity among different studies (*P* < 0.001, *I*^2^ = 89%), and the random effects model was used for analysis. After treatment, 48 h-PAO_2_ of the HFNC group was higher than that of the NIV group; the difference was not statistically significant (SMD = −0.07, 95% CI (-0.67, 0.53), *P* = 0.006) (Figure 7).

### 3.8. Comparison of 48 h-PACO_2_ after Treatment between the HFNC Group and NIV Group

Six studies [16–18, 21–23] compared 48 h-PACO_2_ in the HFNC group and NIV group. The heterogeneity between studies was statistically significant (*P* = 0.04, *I*^2^ = 61%) and was analyzed using a random effects model. After treatment, 48 h-PAO2 in the HFNC group was higher than that in the NIV group; the difference was statistically significant (SMD = −0.36, 95% CI (-0.66, -0.05), *P* = 0.02) (Figure 8).

### 3.9. Comparison of 48 h-pH after Treatment between the HFNC Group and NIV Group

Four studies [16, 18, 21, 23] compared the 48 h-pH of the HFNC group and NIV group. There was no statistically significant difference in heterogeneity among different studies (*P* = 0.67, *I*^2^ = 0%), and the fixed effects model was used for analysis. The results showed that there was a statistically significant difference between the HFNC group and NIV group (SMD = 0.25, 95% CI (0.02, 0.47), *P* = 0.03) (Figure 9).

### 3.10. Comparison of 72 h-PAO_2_ between the HFNC Group and NIV Group after Treatment

Three studies [14, 18, 19] compared 72 h-PAO_2_ between the HFNC group and NIV group. There was no significant difference in heterogeneity among studies (*P* = 0.65, *I*^2^ = 0%), and the fixed effects model was used for analysis. The results showed that there was no significant difference between the HFNC group and NIV group (SMD = 0.08, 95% CI (-0.23, 0.39), *P* = 0.61) (Figure 10).

### 3.11. Comparison of 72 h-PACO_2_ between the HFNC Group and NIV Group after Treatment

Four studies [14, 15, 18, 19] compared 72 h-PACO_2_ in the HFNC group and NIV group. There was no significant difference in heterogeneity between studies (*P* = 0.13, *I*^2^ = 48%), and the fixed effects model was used for analysis. The results showed that there was no significant difference between the HFNC group and NIV group (SMD = −0.10, 95% CI (-0.31, 1.43), *P* = 0.36) (Figure 11).

### 3.12. Comparison of 72 h-pH between the HFNC Group and NIV Group after Treatment

Three studies [14, 18, 19] compared 72 h-pH levels between the HFNC group and NIV group. The heterogeneity between different studies was statistically significant (*P* = 0.002, *I*^2^ = 84%) and was analyzed using a random effects model. The results showed that there was no significant difference between the HFNC group and NIV group (SMD = −0.43, 95% CI (-1.07, 0.21), *P* = 0.18) (Figure 12).

### 3.13. Publication Bias

A total of 12 articles [12–23] were included in this study, and the funnel plot of 24 h-PAO2 and 24 h-PACO_2_ was used to evaluate publication bias. The results show that the funnel plot of the observed index is basically symmetric, and the shape of the funnel plot does not show any obvious asymmetry. The results showed no evidence of publication bias (Figure 13).

## 4. Discussion

Acute exacerbation of COPD is characterized by sudden exacerbation of respiratory symptoms, decreased respiratory function, and poor prognosis [3]. Patients with moderate to severe exacerbations of COPD often develop acute respiratory failure, which often requires emergency department and hospitalization. NIV is recommended as an additional method of treatment for patients with COPD acute progressive exacerbation and respiratory failure [24]. NIV has been shown to reduce intubation rate and improve the survival rate of COPD patients requiring ventilation support, and it is recommended to be used in the treatment of COPD patients with type II respiratory failure [25]. However, NIV has disadvantages, such as reduced comfort and poor interaction and synchronization between patients and ventilators, which are often difficult to identify and manage [26]. In recent years, HFNC has been increasingly applied in stabilizing and aggravating COPD patients [27].

Meta-analysis results of this study showed that PaO_2_ level in HFNC group was higher than that in the NIV group after 12 h and 48 h. The PaCO_2_ level of the HFNC group at 48 h was higher than that of the NIV group. There was no significant difference in 12 h-PACO_2_, 24 h-PAO_2_, 24 h-PACO_2_, 24 h-pH, 48 h-PAO_2_, 72 h-PAO_2_, 72 h-PACO_2_, and 72 h-pH between the two groups after treatment. NIV has been proven to be an effective respiratory support technique that improves gas exchange, reduces the need for intubation in patients with COPD, acute cardiogenic pulmonary edema, and blunt chest trauma, and reduces mortality [28]. Plant et al. [29], in a landmark study involving 236 patients, half of whom received standard therapy and additional NIV, showed that early NIV in COPD patients with mild and moderate acidosis in the common ward resulted in rapid improvement of physiological variables. Reduce the need for invasive mechanical ventilation and in-hospital mortality. NIV in the treatment of acute respiratory failure can deal with abnormal gas exchange and reduce signs of dyspnea and activities of accessory respiratory muscles [30]. However, NIV intolerance is a frequently occurring condition that increases NIV failure rates, intubation rates, and overall mortality [31]. In addition, patients' discomfort and adverse reactions frequently occur in the process of use, such as skin damage, air leakage, and claustrophobia, resulting in poor tolerance of patients.

HFNC is a novel oxygen therapy with good tolerability. HFNC is theoretically suitable for patients with COPD because it can provide a higher airflow, but a relatively low level of FiO_2_ in inhaled air can produce a smaller positive average airway pressure, relieving respiratory distress and reducing respiratory work. HFNC continuously expels carbon dioxide from the upper respiratory tract (flushing dead nasopharyngeal cavities), reducing dead cavities and allowing more efficient alveolar ventilation. The beneficial effects of HFNC include the following: delivery of high flow, better matching of patients' peak inspiratory flow, and finally enabling the implementation of FiO_2_ setting, providing a small amount of positive pressure in the airway to increase end-expiratory lung volume, flushing of nasopharyngeal dead spaces to enhance CO_2_ removal, with good tolerability and comfort [32–35]. Several studies have shown that HFNC improves respiratory work and breathing patterns in patients with acute hypoxic respiratory failure compared with conventional oxygen therapy. Facial skin breakage due to long-term treatment is more common and can increase intolerance to NIV. In addition, the release of warm, moist air through the nostrils avoids the discomfort caused by NIV masks putting pressure on the facial skin, and HFNC is better tolerated than NIV and can be used continuously for longer periods of time.

In summary, the use of a nasal cannula to deliver high-flow heating and humidifying gases at a preset FiO_2_ ratio is an attractive alternative to conventional oxygen therapy and may be an alternative to NIV.

## Figures and Tables

**Figure 1:** Risk of bias summary.

**Figure 2:** Comparison of 12 h-PAO_2_ after treatment between the HFNC group and NIV group.

**Figure 3:** Comparison of 12 h-PaCO2 after treatment between the HFNC group and NIV group.

**Figure 4:** Comparison of 24 h-PAO_2_ after treatment between the HFNC group and NIV group.

**Figure 5:** Comparison of 24 h-PACO_2_ after treatment between the HFNC group and NIV group.

**Figure 6:** Comparison of 24 h-pH after treatment between the HFNC group and NIV group.

**Figure 7:** Comparison of 48 h-PAO_2_ after treatment between the HFNC group and NIV group.

**Figure 8:** Comparison of 48 h-PACO_2_ after treatment between the HFNC group and NIV group.

**Figure 9:** Comparison of 48 h-pH after treatment between the HFNC group and NIV group.

**Figure 10:** Comparison of 72 h-PAO_2_ after treatment between the HFNC group and NIV group.

**Figure 11:** Comparison of 72 h-PaCO_2_ after treatment between the HFNC group and NIV group.

**Figure 12:** Comparison of 72 h-pH after treatment between the HFNC group and NIV group.

**Figure 13:** Funnel plot.

## Data Availability

The simulation experiment data used to support the findings of this study are available from the corresponding author upon request.
